The article "Research Progress on the Relationship between Dietary Patterns and Hyperuricemia" was retracted in 2023. Reasons: signs of a paper mill; suspected computer-generated content; unreliable results or conclusions; concerns about the data.

# Research Progress on the Relationship between Dietary Patterns and Hyperuricemia

**DOI:** 10.1155/2022/5658423

**Published:** 2022-09-17

**Authors:** Tian Long, Liang Liu

**Affiliations:** Department of Clinical Nutrition, Huangshi Central Hospital, Affiliated Hospital of Hubei Polytechnic University, Edong Healthcare Group, Huangshi, Hubei 435000, China

## Abstract

As the final metabolite of purine metabolism, uric acid is critically associated with human health. The serum uric acid level is regulated by diet and the metabolic capacity of the human body. The impaired control of uric acid metabolism and excretion is associated with the increased level of serum uric acid, which ultimately results in hyperuricemia. Hyperuricemia is the “fourth-highest” after hypertension, hyperglycemia, and hyperlipidemia. With progress made in the relationship between diet and hyperuricemia, different dietary patterns and lifestyles have been discussed, such as exercise, the amount intake of meat, seafood, supplements with omega-3 fatty acids, sugar-sweetened soft drinks and energy drinks, and lower-fat-containing foods as well as drinking beer, wine, and spirits in the present article. This study demonstrated that a lower risk of hyperuricemia is substantially correlated with higher baseline adherence to MeDiet, and plant polyphenols can combat hyperuricemia by blocking xanthine oxidase.

## 1. Introduction

### 1.1. The Introduction of Uric Acid

Uric acid was discovered by Carl Scheele (1742–1786). At the same time, Tobern Bergman discovered that uric acid is a major constituent of bladder stones. In the same year, Murray Forbes suggested that both urine and blood may contain uric acid. Alfred Baring Garrod (1819–1909) discovered that the uric acid level is higher in the blood of gout patients. Nobel laureate Emil Fischer (1852–1919) identified uric acid as a purine compound. Studies of uric acid metabolism by isotope tracer techniques have shown that urate overproduction can be detected in about one-third of gout patients [1].

The studies of De Xie have shown that the final product of purine metabolism is uric acid. The uric acid is synthesized by the action of several enzymes, including xanthine oxidase (XO). The enzyme XO catalyzes the final two steps in the conversion of uric acid from purine. The catalytic reaction is hypoxanthine to xanthine and the second catalytic reaction is xanthine to uric acid [2]. As an endogenous antioxidant, uric acid substantially scavenges the free radicals, including monooxyperoxy radicals (ROS) and hydroxyl radicals (OH) [3]. In contrast, uric acid is unable to scavenge the superoxide radical, and uric acid exerts its antioxidant capacity in the presence of ascorbic acid in plasma. Although uric acid is a substantial antioxidant in the extracellular fluid, uric acid acts as a prooxidative agent in the cellular system [2]. In the cellular system, the prooxidative effect of uric acid is regulated by the NADPH oxidase-dependent regulatory pathway. Studies have confirmed that the uric acid level in plasma is considered a circulatory marker of oxidative damage, which is significantly observed in various clinical complications, including ischemia–reperfusion injury, ischemic liver injury, heart failure, chronic atherosclerosis, hyperlipidemia, and diabetes [4–7].

The article "Research Progress on the Relationship between Dietary Patterns and Hyperuricemia" was retracted in 2023. Reasons: signs of a paper mill; suspected computer-generated content; unreliable results or conclusions; concerns about the data.

## 2. Background of Hyperuricemia

Uric acid, the final product of purine catabolism, is mainly catalyzed by the XO enzyme [8], and it is excreted from the body through urine and feces [9, 10]. Uric acid in serum is susceptible to purine- and fructose-rich diets and is synthesized by the catabolism of macromolecules, including DNA, RNA, and ATP. The uric acid is mainly excreted by the kidney, and failure of renal function can also promote the re-elevation of serum uric acid. At the same time, hormones, including estrogen, can augment the excretion of uric acid and it is associated with lowering serum uric acid levels in premenopausal women. Renal vasoconstriction also reduces the excretion of urate. The serum urate level is impaired when the transport system is genetically altered, especially genetic polymorphisms of SLC2A9, which regulates Glut9, affect serum urate levels [11, 12]. When urate production and excretion are unbalanced, serum urate levels also increase significantly [13]. As the name suggests, hyperuricemia refers to an abnormally elevated serum uric acid concentration of >7 mg/dL (416 *μ*mol/L) in men and >6 mg/dL in women, which is considered hyperuricemia [14]. The average levels of serum uric acid have been increasing in many populations over the last century [15]. Epidemiological studies show 170 million patients with hyperuricemia in China, compared with 32.5 million in the United States [16]. Findings from 2009 to 2010 showed that the prevalence of hyperuricemia in the US adult population was approximately 19.3% [17], and its prevalence increased over time [9, 18, 19]. According to NHANES data, the levels of uric acid in the United States significantly increased from 19% in 1988–1994 to 21.5% in 2007–2008 [20]. Results of an epidemiological survey study in the eastern coastal areas of China revealed the prevalence of hyperuricemia which was about 13% in 2008, while it was considered nonexistent in the 1980s. The results showed that the prevalence of hyperuricemia was higher in Oceania countries, including Thailand (Lohsoonthorn et al., 2006), China (Nan et al., 2006), the United States (Zhu et al., 2011), Australia (Nabipour et al., 2011), France (Zalokar et al., 1972), England (Gimeno et al., 2009), New Zealand and Scotland (Sturge et al., 1977), and to a lesser extent in African countries, Malaysia, Turkey, Iran, Saudi Arabia, Philippines, and regions of the Soviet Union (Kuo et al., 2015; Gosling et al., 2014) [21].

The article "Research Progress on the Relationship between Dietary Patterns and Hyperuricemia" was retracted in 2023. Reasons: signs of a paper mill; suspected computer-generated content; unreliable results or conclusions; concerns about the data.

## 3. Complications of Hyperuricemia

Hyperuricemia is associated with gout and various cardiometabolic diseases, especially in type 2 diabetes, coronary artery disease, kidney disease, myocardial infarction, stroke, obesity, atherosclerotic heart disease, hypertriglyceridemia, and other metabolic syndromes [22]. Recent studies suggest that hyperuricemia is critically associated with the risk factor for these diseases [10]. In this article, we substantially discuss this relationship and evaluate the pros and cons of therapeutic interventions (Table 1).

### 3.1. Uric Acid is Associated with Metabolic Syndromes

A 10-year follow-up study showed that high SUA in children (10–15 years) is a crucial predictor of MS events in male subjects [23]. A prospective study evaluating 1,511 men and women aged 55 to 80 initially showed that they were not affected by any MS component. Later follow-up results showed that MS had a significantly higher incidence of hypertriglyceridemia, low high-density lipoprotein (HDL), and Htn [24]. A prospective meta-analysis study with more than 54,000 participants revealed that increased SUA was correlated with an augmented risk of MS and also a causal risk factor for nonalcoholic fatty liver disease (NAFLD) [25].

### 3.2. Chronic Kidney Disease

The kidneys are responsible for excreting 65–75% of uric acid daily, and the gastrointestinal tract is responsible for excreting the remaining 25–35% [26]. Impaired renal excretion is associated with about 90% of hyperuricemias [10]. Also, 60% of patients can develop hyperuricemia in advanced chronic kidney disease (CKD) [27]. Furthermore, CKD is a frequent independent risk factor for developing gout [28]. CKD can be defined as a structural or functional abnormality of the kidney that persists for more than 3 months [29]. These abnormalities included the lower glomerular filtration rate (GFR < 60 mL/min/1.73 m^2^) or the impairment of one or more than one markers of renal failure [29]. CKD is associated with the increasing prevalence of metabolic disease and cardiovascular diseases with an increasing problem of global public health, accounting for approximately 14% of the US population [30]. Over the past two decades, hyperuricemia is critically associated with the risk factor to develop or progress CKD, but its causality remains uncertain. Recent human epidemiological data and experimental evidence from animal models of mild hyperuricemia suggest that soluble serum urate may be directly involved with the pathogenesis of CKD [31, 32].

The article "Research Progress on the Relationship between Dietary Patterns and Hyperuricemia" was retracted in 2023. Reasons: signs of a paper mill; suspected computer-generated content; unreliable results or conclusions; concerns about the data.

### 3.3. Systemic Hypertension

The risk of hypertension increases with age in patients with hyperuricemia [33, 34]. In children, studies discovered that an increased SUA level is substantially correlated to the development and pathogenesis of de novo primary hypertension [35]. A prospective meta-analysis study with 97,824 participants showed a higher level of SUA-predicted systemic hypertension [36]. Of the 118,000 healthy subjects from 40 to 70 years old were diagnosed with the level of SUA in 2002, and developed a quarter with systemic hypertension over the next 10 years. They found that subjects with SUA higher than 3 mg/dL showed a greater risk of developing hypertension. Within the normal range, a higher level of SUA is associated with a greater risk of developing hypertension [37, 62]. One of the important determinants of SUA is the glucose transporter “GLUT9” gene. GLUT9 transports UA. A family study of GLUT9 gene polymorphisms showed that hyperuricemia can lead to systemic Htn [38].

## 4. Dietary Pattern

The important organs, including the liver, muscles, and gut delivered two-thirds of the uric acid load, whereas the other food and drink constituents, including seafood, alcohol, fructose, and purine-rich meats delivered the rest of the uric acid. An important way to lower uric acid is to change patients' diet and lifestyle.

## 5. Diet

Different types of foods contain different amounts of purines. It was previously mistakenly believed that avoiding high-purine foods was the only basis for a proper diet for people with gout. Up-to-date cross-sectional research in China revealed that the augmented prevalence of hyperuricemia is significantly correlated with the intake of a higher amount of wheat products, fresh meat, animal offal, and fish [39]. Researchers studied the association between the intake of higher purine-containing food and protein and the prevalence of hyperuricemia in 3978 men aged 40–74 years and revealed a strong correlation between the intake of seafood and hyperuricemia [40]. In contrast, the intake of soy and soy foods is inversely correlated with the prevalence of hyperuricemia [40]. Moreover, all animal foods are not associated with the risk of developing gout. Such as dairy products with low fat showed a protective effect. Studies have shown that the intake of dairy products, intake of lactose, and supplementation of calcium are inversely correlated with the level of plasma urate [41, 42].

The article "Research Progress on the Relationship between Dietary Patterns and Hyperuricemia" was retracted in 2023. Reasons: signs of a paper mill; suspected computer-generated content; unreliable results or conclusions; concerns about the data.

A population-based meta-analysis indicated that intake of alcohol, meat, and potatoes was significantly correlated with the increased level of serum uric acid, whereas peanuts, skim milk, eggs, cold cereal, butter, brown bread, and noncitrus fruits were correlated with a lower level of serum uric acid [43]. Prospective cohort studies suggest that the individual risk of the patient may represent a critical interaction between unmodifiable factors, including age, sex, ethnicity, and genetic materials, and modifiable factors, including intake of diet, the weight of subjects, and lifestyle. Also, taking the existing information from available the literature, it can be elaborated that intake of meat, drinking of alcohol, seafood, purine-rich food intake, fructose or sugar-sweetened beverages (SSBs) are significantly correlated with increasing the risk of gout, whereas other food and drinking agents, including dairy food, coffee, vitamin C, and cherries were associated with the protection subjects from hyperuricemia and gout [44]. Another study of a 19-item prospective cohort found that the intake of red meat, seafood, alcohol, or fructose is positively correlated with the risk of hyperuricemia and gout. In contrast, other food items, including dairy products, soy food, fruits, and drinking coffee were negatively correlated with the risk of hyperuricemia and gout. It can be correlated with a greater risk of hyperuricemia in women but diminished the risk of hyperuricemia in men [45].

## 6. Plant-Based Diets

Plant-based diets (PBDs; including less animal-food intensive, vegetarian, and vegan diets) attract a growing area of interest in the promotion of physical and environmental health. In chronic non-communicable diseases, a PBD can reduce the risk of morbidity and mortality in patients [46–50].

Several factors, including lower alcohol intake, weight loss, a diet with low purines, and total protein intake, are considered to treat and prevent gout attacks. However, reducing the intake of protein from animal sources will influence the utilization of refined carbohydrates and saturated and trans fats, which will have adverse effects on the cardiovascular system [51]. PBD is primarily centered on vegetables, legumes, grains, whole grains, and many other fruits. The results of a study revealed that the serum concentration of UA was lower in the vegetarian group than that in the nonvegetarian group [51].

## 7. Legumes

Beans are an important component of PBD plant-based dieters [52], are lower in natural fat, and showed a reduced level of the glycemic index. In PBD, beans supplemented a greater percentage of micro- and macronutrients, including dietary fiber, B vitamins, zinc, iron, and other essential minerals. Findings showed that soy foods were a crucial dietary agent which is associated with a longer survival time in older adults [53]. Soy foods are high in the diets of Asian countries, but soy products may increase the risk of gout. However, a prospective cohort study of 63,257 Chinese adults showed that legume-based products, including soy and nonsoy products, were correlated with a decreased risk of gout [70], and soy protein substantially increased the serum UA level. A plant food-rich diet has not been found to influence the risk of hyperuricemia and gout [54]. In their gout management recommendations, the British College of Rheumatology also encourages patients to include soy and plant proteins in their diets, while avoiding high-purine foods [55].

The article "Research Progress on the Relationship between Dietary Patterns and Hyperuricemia" was retracted in 2023. Reasons: signs of a paper mill; suspected computer-generated content; unreliable results or conclusions; concerns about the data.

## 8. Plant Polyphenols

Vegetables and fruits are significantly correlated to reducing the incidence of various diseases such as hypertension, cardiovascular disease, cancer, diabetes, hyperuricemia, and gout [21]. It may be related to the presence of a large number of bioactive components (such as polyphenols) contained in vegetables and fruits [56]. Polyphenols are the most common functional bioactive components, and plant polyphenols can combat hyperuricemia by blocking XO to reduce UA synthesis, inhibit renal reabsorption of urate, and improve UA secretion [57].

## 9. Mediterranean Diet (MeDiet)

MeDiet is defined as a high intake of vegetables, fruits, legumes, nuts, olive oil, and whole grains and an intake of moderate level of poultry, dairy products, and wine. Since MeDiet showed the properties of antioxidant and anti-inflammatory activities [58], it may exhibit the role to reduce the SUA concentration, a crucial independent predictor of cardiovascular disease (CVD) in individuals with a high risk of cardiovascular disease [59]. In a study of 4,449 heart patients, a prospective analysis of older participants with high vascular risk showed that after a median follow-up of 5 years, 756 (24.9%) of 3,037 without hyperuricemia at baseline developed hyperuricemia compared with 964 at baseline. Four hundred twenty-two of those (43.8%) recovered from this condition. A cross-sectional study found an inverse association between the increased levels of adherence to the 14-item MeDiet score and decreased hyperuricemia. This demonstrated that a lower risk of hyperuricemia is substantially correlated with higher baseline adherence to MeDiet [60].

## 10. Recommended Lifestyle with Hyperuricemia Complications

The following health advice is for patients with gout, but also patients with hyperuricemia, cardiovascular disease, obesity, coronary artery disease, metabolic syndromes, hypertension, diabetes, and hyperlipidemia. These recommendations are as follows [61]:

1. Exercise every day to lose weight. Weight loss was used to help reduce SUA in patients; however, the effect of this approach was modest (obese patients with gout lost an average of 7.7 kg over 16 weeks, a mean difference of 1.6 mg/dL SUA).

2. Limited intake of meat, seafood, and supplements with omega-3 fatty acids. Previous studies have revealed that consumption of meat and seafood is critically correlated with the development of hyperuricemia.

3. Intake of limited sugar-sweetened soft drinks and energy drinks is recommended. Intake of fructose is associated with increased SUA, and intracellular fructokinase produces an increased level of local ATP consumption and AMP production from the fructose [17]. It was reported that the supplemented high-calorie fructose (+35% excess energy) with extreme doses (213–219 g/day) substantially increased the level of SUA (mean difference = 0.5 mg/dL).

4. Eating lower-fat-containing foods or nonfat dairy-based products and reducing the intake of food-containing saturated fat, solid fat, and harmful cholesterol had little enforcement on reducing the level of SUA.

5. Cut down on drinking beer, wine, and spirits.

The article "Research Progress on the Relationship between Dietary Patterns and Hyperuricemia" was retracted in 2023. Reasons: signs of a paper mill; suspected computer-generated content; unreliable results or conclusions; concerns about the data.

## 11. Conclusion

This study demonstrated that a lower risk of hyperuricemia is substantially correlated with higher baseline adherence to MeDiet, and plant polyphenols can combat hyperuricemia by blocking xanthine oxidase.

## Figures and Tables

**Table 1:** The relationship between hyperuricemia and dietary pattern.

Diet	Hyperuricemia
Higher purine-containing food and protein	Positive
Soy and soy foods	Negative
Dairy products with low fat	Positive
Alcohol, meat, and potatoes	Positive
Peanuts, skim milk, eggs, cold cereal, butter, brown bread, and noncitrus fruits	Negative

## Data Availability

The data used to support this study are available from the corresponding author upon request.
